The article "Temperature effects on life history traits of two sympatric branchiopods from an ephemeral wetland" was retracted in 2023. Reasons: duplicate publication; unreliable results or conclusions; concerns about the data.

# Temperature effects on life history traits of two sympatric branchiopods from an ephemeral wetland

**DOI:** 10.1371/journal.pone.0179449

**Published:** 2017-06-27

**Authors:** Wan-Ping Huang, Lien-Siang Chou

**Affiliations:** Institute of Ecology and Evolutionary Biology, National Taiwan University, Taipei, Taiwan; Zhejiang University College of Life Sciences, CHINA

## Abstract

Temperature effects on organisms are of multiple scientific interests, such as for their life history performance and for the study of evolutionary strategies. We have cultured two sympatric branchiopod species from an ephemeral pond in northern Taiwan, *Branchinella kugenumaensis* and *Eulimnadia braueriana*, and compared their hatching rate, maturation time, sex ratio, growth of body length, survivorship, clutch size, net reproductive rate *R*_*0*_, generation time T_G_, and intrinsic rate of natural increase *r* in relation to temperature (15, 20, 25 and 30°C). We found that *E*. *braueriana* had a significantly higher temperature-dependent fecundity and intrinsic population growth pattern (*R*_*0*_ and *r*). In contrast, *B*. *kugenumaensis* reproduced much slower than *E*. *braueriana* with much lower *R*_*0*_ (90–100 folds less) and *r* (about 10 folds less) at 15, 20 and 25°C and with a double as long T_G_ at 20 and 25°C. In addition, *E*. *braueriana* increased its chance of hermaphroditic sexual reproductive mode at higher temperature because of a significantly delayed maturation of males from hermaphrodites. In contrast, *B*. *kugenumaensis* showed no significant change in reproductive mode with temperature. This is the first study indicating a significant differentiation in life history parameters of two sympatric branchiopods mediated by temperature.

## Introduction

Temperature is a key factor for growth, development, reproduction, and survival of organisms [1–5]. Various studies have demonstrated that animals could grow or reproduce faster at elevated temperatures. For example, the marine copepod *Calanus finmarchicus* (Gunnerus, 1770) grew faster with elevated respiration rate at higher temperature [2]. The fairy shrimp *Branchinecta lindahli* Packard, 1883 matured faster with increasing temperatures along a latitudinal gradient [5]. The moth *Busseola fusca* (Fuller, 1901) showed smaller clutch size at increased temperature [1]. However, elevated temperature could also cause reduced survivorship. The amphipod *Gammarus pulex* (Linnaeus, 1758) died earlier with increasing temperature at an experimental range of 10–20°C [4].

Temperature also affects animal behavior, interspecific relationships, and niche realization [6, 7]. The hemipteran insect *Anisops sardeus* Herrich-Schaeffer, 1849 ate the larvae of *Anopheles stephensi* Liston, 1901 in a temperature-dependent manner. Its foraging activities increased at elevated temperatures between 20°C to 30°C [6]. Algae are producers and common food for many aquatic invertebrates. The green algae *Scenedesmus obliquus* (Turpin) Kützing, 1833 grew faster at higher temperatures (e.g. 35°C), however, formed smaller colonies (e.g. four-cell colony) especially under *Daphnia* filtrate condition [7]. These evidences showed that temperature could influence the behavior of predators (e.g. *Anisops sardeus*) as well as the colony formation of preys (e.g. algae), affecting interspecific relationships and their niche.

At Siangtian Pond of Yangmingshan National Park, Taipei, Taiwan [8], the fairy shrimp *Branchinella kugenumaensis* (Ishikawa 1895) and the clam shrimp *Eulimnadia braueriana* Ishikawa, 1895 coexisted for a long time. Siangtian Pond, a temporary wetland that is dry for most of the year and becomes water-filled following heavy rainfalls during typhoons [9]. It inundates commonly from June to November with average water temperatures ranging from 21°C to 26°C (see Table A in S1 File for inundation records during the years of 2006–2012). Both species showed spatial niche differentiation in the sympatric pond [8]. The fairy shrimp *B*. *kugenumaensis* exhibited the phenotypic plasticity on growth with presumably optimal resource [9]. From the laboratory culturing experiment, Huang and Chou (2015) found temperature influence on *E*. *braueriana* as it grew faster and died earlier at higher temperatures (25, 30°C) with significantly different developmental time between males and hermaphrodites (the counter sex form from males and capable of producing sperms and eggs by itself) [10]. Therefore, we hypothesize that the temperature can put different effects on growth and reproductive patterns of these two branchiopod species, and may even lead to a niche-differentiation between them.

We investigated the specific niche conditions that enable both branchiopods to co-exist in such a variable environment. Since temperature is an important factor in this habitat, we hypothesize that the performance of life history traits and different reproductive modes depend on temperature. To test this hypothesis, we cultured egg-containing sediments from Siangtian Pond in laboratory mesocosms at four different temperatures (15, 20, 25 and 30°C), recorded the earliest hatching time (EHT), earliest maturation time (EMT), maximum lifespan (MLS), sex ratio (or male percentage), and measured or estimated the growth (body length), survivorship, clutch size, net reproductive rate (*R*_*0*_), generation time (T_G_) and intrinsic rate of natural increase (*r*) of each resulting cohort. Finally, all above life history traits of these two species were compared and interpreted from an ecological as well as from an evolutionary perspective.

## Methods

### Study site

The study site, Siangtian Pond, Yangmingshan National Park, northern Taiwan (25°10’N, 121°30’E) is publicly owned. With the date of 2009/08/31 a valid field license number 20091403 was provided for the present study. In this area are no endangered nor protected species present nor involved in our study (see also field licence–Figure C in S1 File).

### Sample collection

Dormant eggs were collected from the dry surface substrate of Siangtian Pond, Yangmingshan National Park (25°10’N, 121°30’E). Siangtian Pond is a seasonally temporary wetland and inundates after heavy rains mainly during typhoons. The pond can be sometimes 80 m in diameter with a depth of up to 5 m. The water level can fall for about 30 cm per day, keeping the ponds inundated for commonly only 2–3 weeks [8, 9].

Collected substrate with dormant eggs was air dried indoors for more than two weeks. Then the substrate was gently stirred to become homogenous. In laboratory, four temperature trials (15, 20, 25, 30°C) were conducted with 20 replicates each, making 80 cultures in total. Each culture contained 100 g of substrate mud with dormant eggs in a plastic container (3.6 L, 20x12 cm^2^, 15 cm in height), which was covered with 2 L filtered water (Amway eSpring Water Filter, 0.2 μm in mesh size). The photoperiod was set at 14 hours light (50–60 Hz, 14 W) and 10 hours dark [10]. The mesocosms with the collected substrate provided the growth of cyanobacteria and algae within a short period of time.

Mesocosm incubations were carried out at the four temperatures, 15, 20, 25 and 30°C with a daily temperature variation of ±1°C. Each temperature treatment contained 20 independent repeats. After emergence of branchiopod larvae, photos were taken daily from each shrimp. The number of hatching larvae was quite variable, ranging from 30 to 200 per plastic container.

Life history traits of *B*. *kugenumaensis* and *E*. *braueriana* were studied, including hatching rate, earliest hatching time (EHT), earliest maturation time (EMT), maximum lifespan (MLS), sex ratio (or male percentage), body length, number of survivors, clutch size, net reproductive rate (*R*_*0*_), generation time (T_G_), and intrinsic rate of natural increase (*r*). Individuals were photographed and body lengths were measured using the software Image J [11]. The body length from 20 individuals per trial, reared at 15, 20, 25 and 30°C were plotted and fitted to sigmoidal growth curves with constants a1 and coefficients b1 by SPSS (PAWS statistics 18, see Eq 1).

$$\text{Body length}=e^{\left(\text{Constant }\left(\text{a}1\right)\;+\;\frac{\text{Coefficient }\left(\text{b}1\right)}{\text{Day}}\right)}$$ (1)

$$\text{Survival number}=\text{Constant }\left(\text{a}2\right)\text{ x }e^{\left(\text{Coefficient }\left(\text{b}2\right)\text{ x Day}\right)}$$ (2)

Clutch size=Constant (a3)+(Coefficient (b3) x Body length) (3)

$$R_{0}=\Sigma_{\text{EMT}}^{\text{MLS}}\left(\text{Clutch size}\right)(\frac{\text{Effective survival number}}{\text{Maximum number}})$$ (4)

$${\text{T}}_{\text{G}}=\frac{\sum_{\text{EMT}}^{\text{MLS}}\left(\text{Clutch size}\right)\left(\frac{\text{Effective survival number}}{\text{Maximum number}}\right)\left(\text{Day}\right)\;}{\sum_{\text{EMT}}^{\text{MLS}}\left(\text{Clutch size}\right)\left(\frac{\text{Effective survival number}}{\text{Maximum number}}\right)}$$ (5)

$$r=\frac{\text{ln}R_{0}\;}{{\text{T}}_{\text{G}}}$$ (6)

Survival curves were fitted to an exponential model as a function of days (Eq 2). Embryos were counted and the resulting clutch size was linearly regressed to body length according to Eq 3. Then, combined with Eqs 1, 2 and 3, daily clutch size was plotted as a function of days. The net reproductive rate (*R*_*0*_) was acquired by accumulating daily clutch size from the effective survival members (female or hermaphrodite) from EMT to MLS (Eq 4). T_G_ and *r* were further calculated according to Eqs 5 and 6 [12].

### Statistics

The hatching rate (i.e. proportion of mesocosms with hatched individuals) at different temperatures (15, 20, 25, and 30°C) was statistically compared by Chi-square test for independence. All parameters at the specific temperatures (15, 20, 25 or 30°C), including EHT, EMT, MLS, sex ratio, coefficients of body-length growth (b1), coefficients of survivorship (b2), *R*_*0*_, T_G_, and *r*, were statistically examined by ANOVA or Kruskal-Wallis test, depending on the outcomes of a numerical normality test (SPSS, PAWS Statistics 18). The post hoc analysis for parametric testing was conducted using Tukey HSD and LSD. For nonparametric post hoc examination, Nemeny test was performed [13].

## Results

### Hatching

Hatching rate was significantly temperature-related (Table 1, Chi-square test for independence: p = 0.035 for *B*. *kugenumaensis*, p = 0.001 for *E*. *braueriana*, n = 20 for each temperature group). The hatching rate of *B*. *kugenumaensis* ranges 20–65%, significant higher (65% and 50%) at lower temperatures (15, 20°C). However, the hatching rate of *E*. *braueriana* ranged 30–85% and showed highest (85% and 60%) at intermediate temperatures (20, 25°C) (Table 1).

**Table 1:** Life history traits at different temperatures from *B*. *kugenumaensis* and *E*. *braueriana*.

Life history traits	Temperature (°C)				p-value
	15	20	25	30	
*B*. *kugenumaensis*					
Hatch					
Hatching rate (%)	65	50	45	20	0.035
Hatching trials (n)	13	10	9	4	—
Developmental time					
(day, mean SE)					<.001
EHT	4.7 0.7 ^a^	1.6 0.3 ^b^	1.2 0.2 ^b^	1.0 0.0 ^b^	
EMT of female	17.5 1.8	14.8 2.8	15.4 4.2	NA	0.133
EMT of male	16.0 1.2	10.8 1.1	8.4 1.4	NA	<.001
MLS	17.5 1.8	14.8 2.8	15.6 4.2	7.5 2.2	0.133
Sex ratio					0.074
(Male%, mean SE)	51.5 1.8	53.0 1.3	52.4 1.6	49.8 3.7	
Growth curve					
Constant (a1)	1.475	1.970	2.153	1.253	—
Coefficient (b1)	-7.914 ^a^	-4.284 ^b^	-3.707 ^c^	-1.540 ^c^	<.001
Survival curve					
Constant (a2)	44.012	79.796	33.490	23.263	—
Coefficient (b2)	-0.102 ^a^	-0.108 ^b^	-0.108 ^ab^	-0.106 ^ab^	0.013
*E*. *braueriana*					
Hatch					
Hatching rate (%)	30	85	60	30	0.001
Hatching trials (n)	6	17	12	6	—
Developmental time					
(day, mean SE)					
EHT	5.8 1.5 ^a^	2.7 0.2 ^b^	1.6 0.4 ^c^	1.7 0.4 ^c^	<.001
EMT of hermaphrodite	18.3 4.7	11.9 1.3	7.5 0.7 ^X^	5.3 0.6 ^Y^	0.001
EMT of male	18.3 4.7	13.9 1.7	16.4 2.6 ^X^	13.3 2.2 ^Y^	0.759
MLS	21.5 5.9	17.1 2.2	17.8 2.5	19.5 2.8	0.909
Sex ratio					0.889
(Male%, mean SE)	0.4 0.4	0.5 0.3	0.1 0.1	1.4 1.0	
Growth curve					
Constant (a1)	1.328	1.466	1.470	1.504	—
Coefficient (b1)	-9.307 ^a^	-5.671 ^a^	-2.574 ^ab^	-2.216 ^b^	0.001
Survival curve					
Constant (a2)	30.939	69.419	97.752	109.941	—
Coefficient (b2)	-0.044 ^a^	-0.105 ^b^	-0.120 ^b^	-0.092 ^b^	<.001

Different superscript letters (a, b, c) indicated the significant pairwise groups by post hoc analysis.

The capital superscript letters (X, Y) referred to the significant differences between hermaphrodite and male at 25°C (p = 0.007) and 30°C (p = 0.004) respectively.

Abbreviations: EHT, earliest hatching time. EMT, earliest maturation time. MLS, maximum lifespan.

### Developmental time and sex ratio

The developmental time was also related to temperature (Table 1). Individuals of both species hatched significantly earlier with reduced EHT (earliest hatching time) as temperature increased (Kruskal-Wallis test: ps < 0.001). *B*. *kugenumaensis* hatched on day 4.7±0.7 (mean±SE, n = 13) at 15°C, on day 1.6±0.3 (n = 10) at 20°C, on day 1.2±0.2 (n = 9) at 25°C, and on day 1.0±0.0 (n = 4) at 30°C. The EHT of *E*. *braueriana* was on day 5.8±1.5 (n = 6) at 15°C, day 2.7±0.2 (n = 17) at 20°C, day 1.6±0.4 (n = 12) at 25°C, and day 1.7±0.4 (n = 6) at 30°C (Table 1).

Furthermore, both species matured significantly faster upon increasing temperature (Table 1, Kruskal-Wallis test: p < 0.001 for Male *B*. *kugenumaensis*, p = 0.001 for hermaphrodite *E*. *braueriana*). Male *B*. *kugenumaensis* matured on day 16.0±1.2 (mean±SE, n = 13) at 15°C, day 10.8±1.1 (n = 10) at 20°C, and day 8.4±1.4 (n = 9) at 25°C. This fairy shrimp never matured under laboratory control at 30°C. The EMT of hermaphrodite *E*. *braueriana* was on day 18.3±4.7 (n = 6) at 15°C, day 11.9±1.3 (n = 17) at 20°C, day 7.5±0.7 (n = 12) at 25°C, and day 5.3±0.6 (n = 6) at 30°C (Table 1). Moreover, there were significant differences on the EMT between hermaphrodite *E*. *braueriana* and its male at high temperatures as 25 and 30°C (Table 1, Mann-Whitney test: p = 0.007 at 25°C, p = 0.004 at 30°C).

However, the EMT of female *B*. *kugenumaensis* or male *E*. *braueriana* did not show the temperature-dependent pattern (Table 1, Kruskal-Wallis test: p = 0.133 for the former, p = 0.759 for the latter), nor their sex ratios. *B*. *kugenumaensis* is dioecious (two sex forms of male and female) fairy shrimp with about equal sex ratio of 49.8–53.0% (male percentage, the proportion of male number to total) at different temperatures (Table 1, Kruskal-Wallis test: p = 0.787). *E*. *braueriana* is an androdioecious (two sex forms of male and hermaphrodite) clam shrimp with biased sex ratio of 0.1–1.4% at four temperatures under laboratory control (Table 1, Kruskal-Wallis test: p = 0.757).

### Growth measured as body length

The growth curves of body length measurements resulting from four temperature incubations were provided in Fig 1 (20 trials for each temperature group). Both *B*. *kugenumaensis* and *E*. *braueriana* grew faster with significant larger coefficients (b1) as temperature increased (Table 1, also see Table B in S1 File, Kruskal-Wallis test: p < 0.001 for the former species and p = 0.001 for the latter one). The fairy shrimp, *B*. *kugenumaensis*, grew significantly faster when temperatures were above 20°C (Fig 1A, Kruskal-Wallis test: p < 0.001, post hoc analysis: a, b, b, b, denoting the significant pairwise groups for 15, 20, 25, 30°C). The clam shrimp, *E*. *braueriana*, also grew significantly faster at higher temperatures, i.e. 25°C and 30°C (Fig 1B, Kruskal-Wallis test: p = 0.001, post hoc analysis: a, a, ab, b, denoting the significant pairwise groups for 15, 20, 25, 30°C). The body length of *B*. *kugenumaensis* at EMT was about 2.8 mm, 5.4 mm, and 6.7 mm under 15, 20, and 25°C, but not available at 30°C (estimated from EMT of female in Table 1 and growth curves of Fig 1A). The body length of *E*. *braueriana* at EMT was about 2.3 mm, 2.7 mm, 3.2 mm, and 2.9 mm under 15, 20, 25, and 30°C respectively (estimated from EMT of hermaphrodite in Table 1 and growth curves of Fig 1B).

**Fig 1:** Growth curves of body length at different temperatures. A, *B*. *kugenumaensis*. B, *E*. *braueriana*. Different superscript letters (a, b) indicated the significant pairwise groups of different temperatures by post hoc analysis.

### Survival

Although the body length of both species grew faster at higher temperatures, these branchiopods died earlier with decreased survival rate when reared at higher temperatures (Fig 2). The fairy shrimp, *B*. *kugenumaensis* died faster with a larger coefficient (b2) at 20°C than at 15°C (Table 1, Fig 2A, also see Table C Part A in S1 File, ANOVA test: p = 0.013, post hoc analysis: a, b, ab, ab as the significant pairwise groups for 15, 20, 25, 30°C). The clam shrimp, *E*. *braueriana* died earlier with significant larger coefficients (b2) at higher temperature, especially above 20°C (Table 1, Fig 2B, also see Table C Part B in S1 File, ANOVA test: p < 0.001, post hoc analysis: a, b, b, b denoting the significant pairwise groups for 15, 20, 25, 30°C).

**Fig 2:** Survival curves at different temperatures. A, *B*. *kugenumaensis*. B, *E*. *braueriana*. Different superscript letters (a, b) indicated the significant pairwise groups of different temperatures by post hoc analysis.

### Clutch size

The clutch size was presented as a function of body length (Eq 3). It ranged from 23.1 at EMT to 19.8 after EMT in field from *B*. *kugenumaensis*, and 26.4 (at EMT) to 18.8 (post-EMT) in field from *E*. *braueriana*, making the Eq 3 with a3 = 2.6196 and b3 = 1.369 for *B*. *kugenumaensis*, a3 = 13.214 and b3 = 2.1036 for *E*. *braueriana* (Figure A in S1 File). The average daily clutch sizes at different temperatures (15, 20, 25, 30°C) from laboratory cohorts were modeled and plotted as shown in Fig 3. According to the model curves, we found that *B*. *kugenumaensis* produced more eggs at intermediate temperatures like 20 and 25°C (Fig 3A, also see Figure B Part A in S1 File), while *E*. *braueriana* had larger clutch sizes at higher temperature as 30°C (Fig 3B, also see Figure B Part B in S1 File). The clutch size of *B*. *kugenumaensis* at EMT was about 1.2, 3.9, and 3.5 under 15, 20, and 25°C, but not available at 30°C (estimated from EMT of female in Table 1 and daily clutch sizes in Fig 3A). The clutch size of *E*. *braueriana* at EMT was about 5.4, 4.2, 8.2, and 29.8 under 15, 20, 25, and 30°C respectively (estimated from EMT of hermaphrodite in Table 1 and daily clutch sizes in Fig 3B).

**Fig 3:** Daily clutch sizes at different temperatures. A, *B*. *kugenumaensis*. B, *E*. *braueriana*.

### Net reproductive rate (*R*_*0*_)

The net reproductive rate (*R*_*0*_) of *B*. *kugenumaensis* was higher under the middle range of temperatures (20 and 25°C), and was estimated as 0.1±0.1 (mean±SE, n = 13) at 15°C, 0.5±0.3 (n = 10) at 20°C, 0.4±0.2 (n = 9) at 25°C, 0.0±0.0 (n = 4) at 30°C (Fig 4, also see Table D Part A in S1 File). However, there was no significant difference among these four temperature groups (Kruskal-Wallis test: p = 0.242). In contrast, the net reproductive rate (*R*_*0*_) of *E*. *braueriana* was generally much higher than of *B*. *kugenumaensis* (over 20–200 folds, significantly different for all temperatures, by Mann-Whitney test: ps < 0.001 at 15, 20, 25°C, p = 0.008 at 30°C), and significantly increased at higher temperatures, i.e. 19.8±7.4 (n = 6) at 15°C, 11.8±2.1 (n = 17) at 20°C, 73.4±28.1 (n = 12) at 25°C, 297.0±98.5 (n = 6) at 30°C (Kruskal-Wallis test: p = 0.001; post hoc by Nemeny test: a, a, ab, ac denoted the significant pairwise groups for 15, 20, 25, 30°C) (Fig 4, also see Table D Part B in S1 File).

**Fig 4:** Net reproductive rates (*R*_*0*_) at different temperatures. The symbol star (*) indicated significant difference of *R*_*0*_ between *B*. *kugenumaensis* and *E*. *braueriana* (**p < 0.010, ***p < 0.001). Different superscript letters (a, b, c) indicated the significant pairwise groups by post hoc analysis.

### Generation time (T_G_)

The generation time (T_G_) of *B*. *kugenumaensis* was 27.0±0.0 (day, mean±SE, n = 13), 29.8±1.7 (n = 10), and 27.0±0.0 (n = 9) for the groups reared at 15°C, 20°C, and 25°C, respectively, with no significant difference among these three groups (Kruskal-Wallis test: p = 0.264, Fig 5, also see Table E Part A in S1 File). No fairy shrimp reached maturity in the four hatching trials at 30°C (Table 1, sixteen trials were failed in hatching). In contrast, the generation time (T_G_) of *E*. *braueriana* from the four temperature treatments were 20.3±5.3 (n = 6) at 15°C, 14.0±1.5 (n = 17) at 20°C, 11.0±0.8 (n = 12) at 25°C, 10.6±1.2 (n = 6) at 30°C (Fig 5, also see Table E Part B in S1 File), with no significant differences among them (Kruskal-Wallis test: p = 0.252). Comparing the two species, T_G_ of *B*. *kugenumaensis* was significantly higher than that of *E*. *braueriana* at intermediate temperatures (i.e. 20 and 25°C) (Fig 5, Mann-Whitney test: p = 0.431 at 15°C, p = 0.001 at 20°C, p = 0.009 at 25°C).

**Fig 5:** Generation times (T_G_) at different temperatures from *B*. *kugenumaensis* and *E*. *braueriana*. The symbol star (*) indicated significant difference of T_G_ between *B*. *kugenumaensis* and *E*. *braueriana* (**p < 0.010, ***p < 0.001).

### Intrinsic rate of natural increase (*r*)

The intrinsic rate of natural increase (*r*) of *B*. *kugenumaensis* was -0.04±0.00 (mean±SE, n = 13) at 15°C, -0.01±0.01 (n = 10) at 20°C, 0.00±0.01 (n = 9) at 25°C, not available at 30°C (Fig 6, also see Table F Part A in S1 File), with no significant difference between these temperature groups (ANOVA test: p = 0.192). In contrast, the intrinsic rate of natural increase (*r*) of *E*. *braueriana* was 0.17±0.05 (n = 6) at 15°C, 0.21±0.05 (n = 17) at 20°C, 0.32±0.05 (n = 12) at 25°C, 0.50±0.06 (n = 6) at 30°C (Fig 6, also see Table F Part B in S1 File). The *r*-value at the highest tested temperature (i.e. 30°C) was significantly higher than that at lower temperatures, namely 15 or 20°C (ANOVA test: p = 0.010; post hoc by Tukey HSD and LSD test: a, a, ab, b denoted the significant pairwise groups for 15, 20, 25, 30°C). The *r*-values of *B*. *kugenumaensis* were significantly lower than those of *E*. *braueriana* at all three temperature groups in laboratory cultures (t-test: p = 0.024 at 15°C, p = 0.006 at 20°C, p = 0.031 at 25°C).

**Fig 6:** Intrinsic rates of natural increase (*r*) at different temperatures from *B*. *kugenumaensis* and *E*. *braueriana*. The symbol star (*) indicated significant difference of *r* between *B*. *kugenumaensis* and *E*. *braueriana* (*p < 0.050, **p < 0.010). Different superscript letters (a, b) indicated the significant pairwise groups by post hoc analysis.

## Discussion

### Temperature-dependent life history traits

Temperature is a key factor for development and population growth of organisms. We found that several life history traits of both *B*. *kugenumaensis* and *E*. *braueriana* varied significantly with temperature. They grew and matured faster at higher temperatures. In addition, they showed a lower life expectancy with elevated temperature. Similar to most ectotherms that grow faster with increasing temperature [14, 15], the amphipod, *Hyalella azteca* (Saussure, 1858), developed faster as temperature increased from 5°C to 15°C [16]. The house cricket, *Acheta domesticus*, grew faster with more oxygen consumption and earlier metamorphosis from larval instar to adult at 28°C, compared to 25°C [17]. The yellow grapevine mite, *Eotetranychus carpini* (Oudemans), matured faster with higher egg production at elevated temperatures from 15°C to 30°C. Its intrinsic rate of natural increase (or natural exponential growth rate) “*r*” showed maximum levels at 26°C, which was considered as the optimal temperature for this species [14].

### Phenotypic plasticity

The temperature effect on life history traits might result from phenotypic plasticity in physiological change. We found that both *B*. *kugenumaensis* and *E*. *braueriana* grew faster and died earlier with increasing temperature. A possible explanation for a shortened life expectancy at elevated temperature could be the reduced oxygen availability (or hypoxic conditions) [18–21]. Animals usually have high demand of oxygen consumption at high temperature. Both the caridean shrimp *Palaemon peringueyi* (Stebbing, 1915) and the copepod *Pseudodiaptomus hessei* (Mrázek, 1894) increase their respiratory rate with a temperature-increasing manner [22, 23]. To respond to hypoxia at elevated temperatures, several branchiopods increase their cardiovascular and respiratory functions in general [24–29]. The brine shrimp, *Artemia franciscana* Kelloggs, 1906, showed a higher heart beat rate at elevated temperature (32°C) than at lower temperature (24°C) [28]. It increased the hemoglobin synthesis with higher oxygen-binding ability in response to hypoxia furthermore [27]. The tadpole shrimp *Triops longicaudatus* (LeConte, 1846) was reported to use an allosteric control of hemoglobin oligomerization for oxygen saturation [25, 26]. Hemoglobin was shown to hybridize *in situ* in the fat cells of epipodites from thoracopods of the water flea *Daphnia magna* Straus, 1820 [24]. Accordingly, in response to hypoxia or high temperature, *D*. *magna* showed an elevated heart beat rate, thoracopod movement rate, and the production of high-oxygen-affinity hemoglobin [29].

Phenotypic plasticity upon hypoxia was also demonstrated in fish. Juveniles of the Atlantic cod *Gadus morhua* Linnaeus, 1758 lowered their swimming speed upon hypoxia [30]. The gill surface of the African cichlid *Pseudocrenilabrus multicolor* (Schöller, 1903) even increased its gill surface at low-oxygen conditions [31, 32]. This phenotypic plasticity was traded-off by other morphological characters, i.e. the brain mass and the head length [31, 32]. At normoxia, *P*. *multicolor* had enlarged brain and head for a better response in regards to predation or self-protection. While at extreme environmental conditions like hypoxia, this cichlid fish invested more energy in gill filament enlargement to improve oxygen transport for a better aerobic physiology and individual survival.

### Reproductive flexibility

Besides the effects on physiology and survival, temperature also influenced reproduction with respect to sex ratio, clutch size, and presumably the biological fitness of offspring [33]. The water flea *D*. *magna* exhibited a higher sex ratio with male bias at lower temperature (20°C), while more females developed at higher temperature (30°C) [34]. The butterfly *Bicyclus anynana* (Butler, 1879) produced fewer but larger eggs at lower temperature (20°C), while more but smaller eggs at higher temperature (27°C) [35, 36]. In the current study, though *B*. *kugenumaensis* and *E*. *braueriana* did not show the temperature-dependent sex ratio variations, they demonstrated the reproductive flexibility on clutch size and EMT (earliest maturation time). Our clam shrimp *E*. *braueriana* even exhibited the switch of reproduction mode from gonochorism (cross-fertilization between a male and a hermaphrodite) to hermaphroditism (self-fertilization within a hermaphrodite) as temperature elevated. At higher temperature, *E*. *braueriana* produced much more hermaphroditic eggs that provide faster population growth since all emerging individuals could provide offspring themselves [37]. However, hermaphroditism goes along with reduced genetic heterozygosity [38, 39]. Therefore, *E*. *braueriana* might maintain its population at high temperature with hermaphroditism through the trade-off by offspring fitness reduction.

Hermaphroditism of *E*. *braueriana* was conducted mainly when male matured significantly behind hermaphrodite at high temperature. Male *E*. *braueriana* development was denoted by claspers modified from the first two enlarged thoracopods [40, 41]. The hemoglobin expression in *D*. *magna* epipodites of thoracopods [24] suggested the high oxygen requirement for branchiopod appendage development. It was implied that male *E*. *braueriana* developed slowly due to hypoxic conditions at high temperature. The sexual reproduction of *E*. *braueriana* with combination of gonochorism and hermaphroditism at lower temperature, therefore, might be traded-off by hermaphroditism alone at higher temperature when clasper development is much slower and offspring fitness is presumably reduced from less genetic diversity.

### Temperature-adapted niche-differentiation

In this study, we showed differences in temperature adaptation for life history traits between two sympatric branchiopods, especially their reproductive modes and population growth. Individual productivity refers to net reproductive rate (*R*_*0*_). Population growth is best reflected by intrinsic rate of natural increase (*r*). The clam shrimp, *E*. *braueriana*, showed significant differences in both *R*_*0*_ and *r* at higher temperatures as 25 and 30°C, indicating its optimal temperature at 25–30°C. However, the other sympatric branchiopod in Siangtian Pond, *B*. *kugenumaensis*, showed highest *R*_*0*_ and *r* at lower range (15–25°C). These two sympatric branchiopod species, therefore, demonstrated a temperature-adapted niche-differentiation on individual reproduction and population growth. It is in accordance with the studies in Austria [42], Hungary [43], Yugoslavia [44], and Australia [45] that anostracans (fairy shrimps) are rather cold-adapted temperate water branchiopods favoring 5–15°C [45], whereas *Eulimnadia* sp. belongs to a group of warm-adapted branchiopods preferring 20–40°C [45].

### Evolution of breeding system

Androdioecy is an evolutionarily transitional breeding system between monoecy and dioecy [46, 47]. Monoecious species (composed of hermaphrodites) produce offspring by hermaphroditism (self-fertilization) within themselves, e.g. *Limnadia lenticularis* (Linnaeus, 1761) [48], which has reduced genetic diversity upon extreme inbreeding situation but is advantageous for colonization [49, 50]. Dioecious organisms, in contrast, have relieved inbreeding and elevated fitness by gonochoric reproduction (cross-fertilization) between males and females [37], e.g. *Lepidurus apus lubbocki* Brauer, 1873 [48]. Many *Eulimnadia* species are androdioecious animals composed of few males and majority of hermaphrodites [46]. They reproduce by gonochorism and/or hermaphroditism depending on conditions. At harsh environment (e.g. ephemeral wetland) or in very small population (i.e. hard to encounter males for crossing), hermaphroditism is more advantageous with reproductive assurance than gonochorism [46, 47]. However, males are stable in some percentage for these populations to be evolutionarily maintained [51–53]. In the present study, these two sympatric branchiopod species showed significant differences in generation time (T_G_) at 20°C and 25°C. The clam shrimp *E*. *braueriana* showed only half T_G_ of the fairy shrimp *B*. *kugenumaensis*. This implies a faster evolutionary rate [54] of the androdioecious *E*. *braueriana* than the dioecious *B*. *kugenumaensis*. Androdioecious breeding system contributes to a tactic reproductive strategy in response to dynamic and unpredictable environment, adding the androdioecious *E*. *braueriana* with more competitive strength in natural niche. Therefore, the coexistence of dioecious (*B*. *kugenumaensis*) and androdioecious (*E*. *braueriana*) breeding system might provide a notation of evolutionary balance from niche differentiation between these two branchiopod populations.

### From laboratory to field

This study presented the contrasting life history characteristics and population growth of *B*. *kugenumaensis* and *E*. *braueriana* under different temperature regimes in laboratory. Our result implies a temperature-adapted niche-differentiation and reproductive strategies between these two sympatric branchiopods. In addition, comparing with field observation (Huang’s unpublished data), these two species grew larger (1–7 folds from *B*. *kugenumaensis*, 1–3 folds from *E*. *braueriana*), matured faster (2–5 days earlier from *B*. *kugenumaensis*, 3–10 days earlier from *E*. *braueriana*), and reproduced more (3–35 folds from *B*. *kugenumaensis*, 1–10 folds from *E*. *braueriana*) in field than in laboratory. Therefore, some other factors in addition to temperature (e.g. dissolved oxygen) might be involved.

## Conclusion

Life history traits of the co-existing dioecious fairy shrimp *B*. *kugenumaensis* and the androdioecious clam shrimp *E*. *braueriana* from Siangtian Pond in northern Taiwan were studied here. This pond shows slight seasonal water temperature variations. In laboratory cultures at 15–30°C, temperature-differentiation has its significant effect on fecundity and population growth. *B*. *kugenumaensis* showed optimal net reproductive rate (*R*_*0*_) and intrinsic rate of natural increase (*r*) at lower temperatures (i.e. 15–25°C) and *E*. *braueriana* conversely at higher temperatures (i.e. 25–30°C). We suggest that this temperature variation in life history traits relates to their sexual reproduction, i.e. dioecious *B*. *kugenumaensis* reproduced only by gonochorism at lower temperatures (i.e. 15–25°C); while the androdioecious *E*. *braueriana* laid both gonochoric and hermaphroditic eggs at lower temperatures (i.e. 15–20°C), and showed a switch to hermaphroditic egg production as temperature elevated to 25–30°C. This is the first study demonstrating a potential niche-differentiation related to temperature, which affects the reproduction and life history performance of two sympatric wetland branchiopods. More direct (e.g. hemoglobin expression and oxygen-binding affinity) and indirect (e.g. physico-chemical oxygen capacity, development of pathogenic microbes, food availability) factors in addition to temperature need further studies in future. This may also allow a better understanding of niche-differentiation mechanisms between these two sympatric branchiopods from an ephemeral wetland.

## Supporting information

S1 File **Table A. Inundation information of Siangtian Pond, Yangmingshan National Park, Taipei, Taiwan, from 2006 to 2012**. The record of accumulated rainfall came from Central Weather Bureau of Taiwan. The water temperature was calculated as mean±SE from sampling days (n). **Table B (for** Table 1 **and** Fig 1**). Constants (a1) and coefficients (b1) for the sigmoidal growth curves of body length at different temperatures**. A, *B*. *kugenumaensis*. B, *E*. *braueriana*. **Table C (for** Table 1 **and** Fig 2**). Constants (a2) and coefficients (b2) for the exponential survival curves at different temperatures**. A, *B*. *kugenumaensis*. B, *E*. *braueriana*. **Table D (for** Fig 4**). Net reproductive rates (*R***_***0***_) **at different temperatures**. A, *B*. *kugenumaensis*. B, *E*. *braueriana*. **Table E (for** Fig 5**). Generation times (T**_**G**_) **at different temperatures**. A, *B*. *kugenumaensis*. B, *E*. *braueriana*. **Table F (for** Fig 6**). Intrinsic rates of natural increase (*r*) at different temperatures**. A, *B*. *kugenumaensis*. B, *E*. *braueriana*. **Table G (for** Fig 4 **and S6 Table). Multiple comparisons for net reproductive rates (*R***_***0***_**) from *E*. *braueriana* using Nemeny test as post hoc analysis. Table H (for** Fig 6 **and Table H). Multiple comparisons for intrinsic rates of natural increase (*r*) from *E*. *braueriana* using Tukey HSD and LSD test as post hoc analysis (SPSS, PAWS Statistics 18). Figure A (for** Eq 3**). Linear relationship of clutch sizes and body lengths for** Eq 3. A, *B*. *kugenumaensis* (n = 241). B, *E*. *braueriana* (n = 602). **Figure B Part A (for** Fig 3A**). Daily clutch sizes at different temperatures from *B*. *kugenumaensis***. X-axis: day. Y-axis: clutch size. **Figure B Part B (for** Fig 3B**). Daily clutch sizes at different temperatures from *E*. *braueriana***. X-axis: day. Y-axis: clutch size. **Figure C Field license**. A, Number: 20091403. B, Date: 2009.08.31. C, Studying site: Siangtian Pond, Yangmingshan National Park. D, Studying goal: life history traits of branchiopods in Siangtian Pond.
(DOCX)
